RETRACTED

# Effect of Narrative Nursing Combined with Thinking Map Health Education on Parturient Self-Efficacy and Neonatal Nursing Ability

**DOI:** 10.1155/2022/8466797

**Published:** 2022-05-26

**Authors:** Yan Wang, Yan Xu, Jingjing Li

**Affiliations:** Obstetrics Department of the First People's Hospital of Lianyungang City, Lianyungang 222001, Jiangsu Province, China

## Abstract

The motivation behind this study is to explore the influence of narrative nursing combined with thinking map health education on parturient self-efficacy and neonatal nursing ability. To verify this claim, we have selected 60 parturients who were treated in the hospital from February 2019 to April 2021. Moreover, these patients were randomly assigned to control and study groups. The former received narrative nursing, and the latter received narrative nursing combined with thinking map health education. The nursing satisfaction, maternal and neonatal nursing ability, maternal health knowledge awareness score, maternal self-efficacy, anxiety, and depression scores were compared. Initially, we have compared the nursing satisfaction: in the study group, 22 cases were satisfied, 8 cases were basically satisfied, and 0 cases were dissatisfied, and the satisfaction rate was 100.00%; in the control group, 12 cases were satisfied, 14 cases were basically satisfied, and 4 cases were dissatisfied, and the satisfaction rate was 86.67%. The nursing satisfaction in the study group was higher compared to the control group (*P* < 0.05). Secondly, we compared the mastery of neonatal nursing ability. The study group mastered the relevant knowledge of neonatal nursing in 23 cases, basically mastered 6 cases, and did not master 1 case, with a mastery rate of 96.67%. The control group mastered the knowledge of neonatal nursing in 12 cases, basically mastered 10 cases, and did not master 8 cases with a mastery rate of 73.33%. In the comparison between the two groups, the mastery of neonatal nursing ability in the study group was higher compared to the control group (*P* < 0.05). Considering the scores of maternal health knowledge, the scores of neonatal basic nursing, physiological characteristics, breastfeeding methods, environmental nursing knowledge, vaccination, and physical examination requirements in the study group were higher compared to the control group (*P* < 0.05). In the comparison of maternal self-efficacy, the total scores for promoting development, health care, safety, feeding, and self-efficacy in the study group were significantly higher compared to the control group (*P* < 0.05). Finally, we compared the scores for anxiety and depression. Before nursing, there exhibited no significant difference (*P* > 0.05). After nursing, the anxiety and depression scores decreased. Furthermore, the anxiety and depression scores of the study group were lower compared to the control group (*P* < 0.05). In the health education of primary parturient, the adoption of narrative nursing combined with thought guiding schema can enhance the level of nursing satisfaction and self-efficacy, strengthen the nursing ability of primiparas and the awareness rate of health knowledge, and reduce the occurrence of a maternal bad mood, which is more in line with the requirements of parturient.

RETRACTED

## 1. Introduction

Pregnancy and delivery are normal physiological processes for women [1]. In recent years, with the continuous enrichment of people's access to knowledge, their concept of health has changed significantly than before. In this context, people pay more attention to the health education of parturients, especially the first parturient. As the direct caregivers of newborns, the concept, cognition, and nursing behavior of newborns are closely related to the growth and development of newborns [2]. Pregnant women are prone to obvious changes in their psychological state due to the influence of hormone secretion, appearance changes, and other factors during pregnancy. In the postpartum stage, pregnant women may have negative emotional problems again due to failure to adapt to changes in identity, physical discomfort, lack of perinatal knowledge, and other factors [3]. Negative emotion will not only affect their own health but affect their child-rearing behavior. Self-efficacy is a subjective judgment of individuals that they can successfully carry out a certain achievement behavior. There is a close relationship between a successful experience and individual self-efficacy. If individuals can obtain successful experiences, they can enhance their self-efficacy level. Some studies have indicated that mothers with prenatal parenting experience will have higher parenting self-efficacy after delivery [4]. The parenting efficacy of parturient women before delivery mainly comes from direct experience, indirect experience, and other aspects. Direct experience is the personal experience learned by parturients in the process of child-rearing and operation, and it is the most effective way to enhance the effectiveness of parturient parenting. With regard to multiparturient women, most primary parturients lack direct experience in parenting, and they have less access to professional perinatal knowledge, which brings about the urgent need for this group to learn health education knowledge of neonatal nursing [4]. To enhance their parenting efficiency, health education is a planned, organized, and systematic social education activity. The combination of two different health education models can effectively carry out health education for parturient women and effectively promote their parenting efficiency and neonatal nursing ability [5]. Bedside, care for mothers and infants helps strengthen the rapid growth of maternal and family members' ability to care for newborns [6]. A standardized education path can promote the mastery of nursing knowledge and the improvement of the nursing ability of parturients and newborns [7]. Therefore, it is of practical significance to study the effects of different health education models on parturient self-efficacy and neonatal nursing ability. It has a certain practical significance to enrich their knowledge reserve, promote role adaptation, and strengthen the level of parturient women.

RETRACTED

Health education is utilized primarily to guide people in such a way to form a correct concept of health, which is based on the knowledge-trust-action theory and COX health behavior interaction model, through knowledge to strengthen awareness to change action [8]. Nowadays, a variety of health models, such as small lectures, personalized health education, and quality control circle, are carried out in various departments. In obstetrical nursing, health education methods such as oral education, classroom for pregnant women, and personalized health education are generally adopted, but the mode is monotonous, the content of propaganda is numerous and disorganized, and it is not easy for parturients to remember [9]. Pregnant women's school needs pregnant women to travel back and forth between the family and the teaching site, which is time- and labor-consuming, and each pregnant woman has a different degree of mastery, so the instructors are unable to explain the actual situation of the pregnant women. Although personalized health education is comprehensive and does not need parturients to travel back and forth, with a great deal of knowledge, nurses need to collect, evaluate, and intervene in maternal information constantly [8]. Therefore, it is very important to explore the mode of health education for parturients undergoing cesarean section. In China, mind mapping is mostly employed in course teaching and has achieved good results, but its application in nursing management, teaching, clinical, and other aspects is still in its infancy. However, studies have confirmed the role of mind mapping in the practice of health education [9]. It is believed that mind mapping can help patients with lung cancer develop a reasonable way of health education and provide patients with better diagnoses and treatments. In Zhang Lei's research, the use of mind mapping effectively promoted the triage accuracy of junior nurses for acute abdomen but also enhanced work efficiency [10]. Most nursing scholars take the significance of narrative nursing as the starting point and find that narrative nursing can enhance the negative emotion of breast cancer patients undergoing chemotherapy, promote their confidence in fighting the disease, and strengthen their quality of life [11]. However, the research on the application of narrative nursing combined with thinking map health education in parturient self-efficacy and neonatal nursing ability has not been reported. In order to promote the parturient self-efficacy and neonatal nursing ability, we should face it with a positive attitude and enhance the parturient self-efficacy and neonatal nursing ability, and further research is needed.

RETRACTED

To address these issues, which are described above, we have focused our attention on finding a way to observe the effect of narrative nursing combined with thinking map health education on parturient self-efficacy and neonatal nursing ability. Experimental studies were carried out to verify the authenticity of our claim, and the results showed the idea is convincing.

The remaining manuscript is arranged as given below.

Selection and rejection procedures of the patients along with generalized information are discussed in the subsequent section.

## 2. Patients and Methods

### 2.1. General Information

Sixty parturients were treated in the hospital from February 2019 to April 2021. The patients were randomly assigned to the control group and the study group. The former received narrative nursing, and the latter received narrative nursing combined with thinking map health education. In the control group, the age was 21–44 years old, with an average of (32.91 ± 1.33) years, and in the study group, the age was 20–45 years old, with an average age of (32.96 ± 3.42) years. There was no statistical significance in the general data. This study was permitted by the Medical Ethics Association of our hospital, and all patients noticed informed consent.

#### 2.1.1. Inclusion Criteria

1. At the end of 37–42 weeks of pregnancy, elective cesarean section parturients with indications for a cesarean section
2. Between 21 and 40 years of age
3. The growing gestational age of healthy delivery of newborns (37–42 weeks)
4. Families with informed consent and voluntary participation in the study
5. Reading ability and ability to communicate with others

#### 2.1.2. Exclusion Criteria

1. Pregnant women who have serious heart, liver and kidney diseases, and malignant tumor diseases
2. Pregnant women who have gestational hypertension, gestational diabetes, and so on
3. Pregnant women have infectious diseases such as AIDS, syphilis, hepatitis, and so on
4. People with mental illness
5. One of the main family caregivers of the husband and wife who has neonatal nursing experience and is a sister-in-law
6. Those whose families failed to care or withdraw automatically during the intervention
7. Parturients who had serious maternal and infant complications during the intervention and could not continue to undergo the trial
8. Those whose nursing effect could not be determined and whose data were incomplete

RETRACTED

### 2.2. Treatment Methods

The control group received narrative nursing: the place of intervention in the hospital was mostly in the ward specifically when they were alone or some patients in good condition were invited to the demonstration classroom for intervention. The intervention time was between 2:00 p.m. and 5:00 p.m. to obtain the consent of the patients and try not to affect the normal treatment and the rest of the patients. The intervention time for discharge and recuperation is between 2:00 p.m. and 6:00 p.m., depending on the patient's condition. Through a sincere attitude to gain the trust of patients, take open-ended questions to encourage patients to tell their own stories and fully express their inner thoughts; each intervention time is controlled within the 40 min.

The study group received narrative nursing combined with thought map health education; narrative nursing was the same as the control group; and the details of mind map health education were as follows: (1) after the health education content and mind map complement each other into PPT, the group members were uniformly trained for about 60 minutes; the specific contents were as follows: an overview of mind map and how to use a mind map to explain health knowledge to patients. The team members are required to master the content of the mind map and be able to carry out health education for the patients. The head nurses and researchers assess the members. The members' assessment scores of more than 90 points are qualified, and the members of this research group all pass at one time. (2) On the day, the parturient was admitted to the hospital; the researchers informed her of the basic situation of the department, including the canteen, hot water room, and the location of the doctor's office; informed the director of obstetrics and gynecology, attending physician, head nurse, and responsible nurse; and informed the department to check the fetal heart rate at 9:00, 11:00, 15:00, and 19:00 every day, the time of oxygen inhalation, methods, and matters needing attention. (3) On the first day after admission, the researchers carried the mind map to the bedside of the patients, carried out mind map health education to the parturient, explained the knowledge points at different levels, and focused on the items to be known before operation and postpartum attention. We apply mind mapping to pregnant women. Because the pregnant women are weak 24 hours after operation, and we need to explain it to the pregnant women and their main caregivers together. Mind mapping was used to make parturients and their caregivers know the indicators that need to be observed and the method of lying position after the operation. (4) After the operation, the parturients were sober under anesthesia and tolerated painless body; continued to carry out mental map health education for her, focusing on postpartum exercise, postpartum diet, and general nursing of newborns; and made use of the advantages of graphic, organized, and logical mind mapping to let parturients know the activities of each stage within 48 hours after delivery. It mainly includes the dietary methods and matters needing attention within four weeks after delivery, as well as the general nursing of newborns, and teaches parturients to view their own nursing and neonatal nursing contents through mind mapping tips. Nurses instruct parturients and their families to operate after on-the-spot demonstration. (5) Mind map health education was given to parturients again one day before discharge, focusing on the knowledge of postpartum diseases, other diseases, and neonatal-related diseases. Meanwhile, the researchers also give guidance to the maternal families, making use of the intuitive and hierarchical advantages of mind mapping to enable pregnant women to grasp the causes of postpartum diseases and newborns, specific clinical manifestations, and how to prevent and nurse, and teach parturients to check whether there are disease manifestations and specific nursing methods through mind mapping. During the whole process, the nurse explains each question in detail to the parturient from top to bottom by using the pictorial mind map. If the parturient has other questions, she can also ask questions in time, and the nurse can give timely guidance. Let the parturient remember for 3–5 minutes after each explanation and ask questions on the spot to deepen the memory, about 30 minutes at a time. (6) The WeChat group was set up by the head nurse after discharge, and the researchers added the families of the discharged experimental group to the “mind map nursing mother group of XX Medical University” so that the WeChat group could effectively guide puerperal women and education during the long-distance puerperal period. The researchers sent the mind map to the group, and the pregnant women raised relevant questions in the group in time, such as “do you need to take the child along with the postpartum examination?” and “why do the children never have enough to eat?” At the end of the 42-day puerperal period, the EPDS scale scores, postpartum diseases, and the incidence of neonatal diseases were compared.

RETRACTED

### 2.3. Observation Index

#### 2.3.1. Satisfaction

The self-made questionnaire of nursing satisfaction of parturient women was adopted, which included satisfaction with nurses' attitude, nursing staff's technology, and health education, which was assigned into three options: satisfaction, basic satisfaction, and dissatisfaction. The day of discharge was taken as a fixed period of time to carry out the evaluation, and the nursing satisfaction survey scale was issued for all the parturients in the four groups, and the nursing staff were evaluated by issuing a star nurses' questionnaire. Evaluation standard of nursing satisfaction: nurses follow the nursing operation procedure; the nursing effect is good; the nursing attitude to the parturient is mild; they are praised by the parturient; and they have a strong sense of responsibility for satisfaction, and the nursing procedure is relatively standardized and the nursing effect is good. Nursing attitude is well, without any complaint as basic satisfaction; nursing operation is not standard, which leads to disputes between nursing and parturient; and poor nursing attitude is not satisfactory. Total satisfaction is the sum of satisfaction and basic satisfaction.

#### 2.3.2. Neonatal Nursing Ability

Using the self-made neonatal nursing ability questionnaire, this part includes: on the day of discharge, two medical staff jointly evaluated their neonatal nursing skills and knowledge. It is assigned into three cognitive levels: mastery, basic mastery, and nonmastery. Questionnaire and face-to-face Q & A were employed to observe and compare the knowledge of neonatal basic nursing, physiological characteristics, breastfeeding methods, environmental nursing knowledge, and vaccination and physical examination requirements of the four groups. Mastery rate = (number of mastery cases + basic mastery cases)/total number of cases *∗* 100%.

#### 2.3.3. Awareness Rate of Maternal Health Knowledge

tThe self-made questionnaire based on “Nursing Knowledge of Caesarean Section,” “Nursing of Obstetrics and Gynecology,” and “Pediatric Nursing” was compiled by researcher mentor, head nurse, and researcher himself and Goossens et al. [12]. Through expert letter inquiry, it is considered that the questionnaire can reflect the variables to be measured and accord with the principle of questionnaire compilation. The content validity coefficient is 0.93, and the reliability is 0.83. It can be considered that the reliability and validity of this knowledge questionnaire are good. The questionnaire included 25 items in the 2 dimensions of maternal self-care and neonatal nursing, with a total of 100 points. Around 25–50 points indicated that the scores of maternal and infant nursing knowledge were less; 50–75 points indicated that the scores of maternal and infant nursing knowledge were medium; and 75–100 points indicated that the scores of maternal and infant nursing knowledge were higher. The higher the score, the better the parturient's mastery of maternal and infant nursing knowledge during puerperium.

RETRACTED

#### 2.3.4. Self-Efficacy

In 2006, Prasopkittikun developed SICS to measure the parenting self-efficacy of mothers aged 0–12 months [13]. In 2009, Zang Shaomin translated the table into Chinese [14]. There are 42 items in 5 dimensions of SICS, which are the promotion of development (14 items), health care (13 items), safety (5 items), feeding (8 items), and comprehensive evaluation (2 items). The average content validity coefficient of all the items in the Chinese version of SICS is 0.98, and the score of each item is 0–100. Zero indicates no confidence at all; 50 indicates moderate confidence; and 100 represents complete confidence. The 42 items were all positive scores; the total score of 42 items was assigned by 42; and the total score was between 0 and 100. The higher the score, the better the parenting self-efficacy of the mother.

#### 2.3.5. Mental Health Score

The anxiety status of the parturient was evaluated by the self-rating anxiety scale (SAS), which was compiled by W. K. Zung in 1971 [15]. It has been employed as a self-assessment tool to understand anxiety symptoms in counseling clinic and can accurately reflect the subjective feelings of patients with anxiety tendencies. SAS score >50 is adopted as the criterion for judging primipara with bad mood. SAS has a total of 20 items, using a 4-grade score to assess the frequency of symptoms. The criteria are as follows: “1” means never; “2” is rare; “3” is more; and “4” is all the time. Patients were asked to check the appropriate options according to their actual feelings in the last week. After the evaluation, the scores of 20 items were added, and we reverse calculate items 5, 9, 13, 17, and 19, that is, the crude score (raw score, *x*) was converted, *y* = int (1.25*x*), and the standard score (index score, *y*) was obtained.

Self-rating depression scale (GDS) is employed to evaluate the depression status of parturients, and it is a special depression screening scale, which was created by Zung in 1965 [16]. The scale is widely adopted in depression screening and has good reliability and validity, and studies demonstrate that the Chinese version of GDS has satisfactory reliability and validity, with Cronbach's *α* coefficient of 0.82 and a test-retest reliability coefficient of 0.81–0.92 in 2 weeks. The GDS score >52 was regarded as the criterion for judging the first parturient with a bad mood. The table has a total of 20 items and uses a 4-grade score to assess the frequency of symptoms. The criteria are as follows: “1” means no or little; “2” is a small part of the time; “3” is a considerable amount of time; and “4” is most of the time. It is suggested that 52 points should be used as the boundary score of depression according to different research purposes. The general criteria are as follows: ≤52 points as normal and no depression, 53–62 points as mild depression, and ≥63 points as moderate and severe depression.

RETRACTED

### 2.4. Statistical Analysis

The mathematical statistics software SPSS 24.0 was employed for statistical analysis; the mean ± standard deviation was adopted for statistical description; the *t*-test was employed for comparison of measurement data between groups; and the chi-square test was adopted for comparison of counting data between groups. Bilateral tests were employed in all statistical tests, and when *P* < 0.05, the difference exhibited statistically significant.

## 3. Results and Discussion

### 3.1. Comparison of Nursing Satisfaction

First of all, we compared the nursing satisfaction: in the study group, 22 cases were satisfied, 8 cases were basically satisfied, and 0 cases were dissatisfied, and the satisfaction rate was 100.00% in the study group; in the control group, 12 cases were satisfied, 14 cases were basically satisfied, and 4 cases were dissatisfied in the control group, and the satisfaction rate was 86.67%. The nursing satisfaction in the study group was higher compared to the control group (*P* < 0.05). All the data results are indicated in Figure 1.

Secondly, we compared the mastery of neonatal nursing ability. The study group mastered the relevant knowledge of neonatal nursing in 23 cases, basically mastered 6 cases, and did not master 1 case, with a mastery rate of 96.67%. The control group mastered the knowledge of neonatal nursing in 12 cases, basically mastered 10 cases, and did not master 8 cases, and the mastery rate was 73.33%. In the comparison between the two groups, the mastery of neonatal nursing ability in the study group was higher compared to the control group (*P* < 0.05). All the data results are indicated in Figure 2.

Thirdly, we compared the scores of maternal health knowledge. The scores of neonatal basic nursing, physiological characteristics, breastfeeding methods, environmental nursing knowledge, vaccination, and physical examination in the study group were higher compared to the control group (*P* < 0.05). All the data results are indicated in Table 1.

RETRACTED

### 3.2. Comparison of Maternal Self-Efficacy

Then, we compared maternal self-efficacy. The total scores of developments, health care, safety, feeding, and self-efficacy in the study group were significantly higher compared to the control group (*P* < 0.05). All the data results are indicated in Table 2.

### 3.3. Comparison of Anxiety and Depression Scores

Finally, we compared the scores of anxiety and depression. Before nursing, there exhibited no significant difference (*P* > 0.05). After nursing, the anxiety and depression scores of the two groups decreased. Moreover, the anxiety and depression scores of the study group were lower compared to the control group (*P* < 0.05). All the data results are indicated in Table 3.

## 4. Discussion

With the rapid development of the global economy, the social status of women in China is gradually rising, but the high requirements of education and the great challenges faced by the society also bring heavy pressure on women, resulting in the phenomenon of late marriage and late childbearing [17]. With the significant increase in the number of older and high-risk pregnant women, the rate of the cesarean section also increased sharply [18]. The World Health Organization recommends that the rate of the cesarean section should be less than 15%, while the rate of cesarean section in China is as high as 54% [19]. The cesarean section has always been a controversial mode of delivery; researchers believe that cesarean section should be carried out under the premise of cesarean section indication to ensure maternal and infant safety, but in the absence of absolute cesarean section indication, the cesarean section does more harm than good [20]. There are more complications in cesarean section than in natural delivery, such as postoperative knife pain, postpartum hemorrhage, and wound pain affecting successful lactation. The health care of women and children has always been the focus of public health, but the development of maternal and child health is not optimistic. As of 2010, the number of maternal deaths caused by pregnancy or childbirth complications is still as high as 287,000, and most of them occur in developing countries [21]. Some studies have pointed out that the causes of maternal death include not only medical factors such as postpartum hemorrhage and amniotic fluid embolism but also social factors such as puerperal infection caused by unreasonable hygiene, malnutrition caused by lack of dietary knowledge, and postpartum depression caused by failure to adapt to new roles [22]. In 2013, as many as 2.8 million babies worldwide died within one month after birth, accounting for about 44% of the deaths of children under the age of five. Parturients are new mothers and lack parenting experience; improper nursing may cause neonatal pneumonia, diarrhea, asphyxia, and even death. Thus, it can be seen that it is imperative to effectively enhance maternal and infant nursing knowledge and reduce postpartum complications [23].

RETRACTED

Health education is to guide people to establish a correct concept of health, which is based on the knowledge-trust-action theory and COX health behavior interaction model, through knowledge to strengthen awareness to change action [24]. Nowadays, a variety of health models, such as small lectures, personalized health education, and quality control circle, are carried out in various departments. Mind map, also known as a brain map, is created by TonyBuzan, an Englishman [24, 25]. It uses the expression method of the combination of pictures and words to transform boring and numerous words into pictures that are well organized and easy to understand so that people can memorize relevant knowledge effectively [24]. Some studies have proved that the right brain is in charge of images, colors, overall concepts, and so on, while the left brain is responsible for numbers, logic, and so on, and mind mapping can well combine the left and right brains, which is more conducive to the memory of knowledge [25]. Mind mapping has the capability to assign the disordered and complicated knowledge points to different levels and radially present it in a concise language specifically by highlighting the key points. In clinical nursing, nurses explain the contents of disease-related health education to patients from top to bottom and from primary to secondary according to the content of the mind map [26]. It can not only avoid the omission of knowledge points caused by busy work or low-seniority nurses' lack of professional knowledge but also make patients understand the relevant knowledge faster and better. The mind map was employed to carry out health education for parturient women undergoing cesarean section, in order to make parturients better master maternal and infant nursing knowledge. Likewise, it is used to improve the level of knowledge, enhance maternal confidence in child-rearing, reduce the incidence of postpartum depression and puerperal complications and neonatal diseases, provide some data support for clinical nursing health education, and provide a reference for health education of other diseases [26, 27].

RETRACTED

Narratology is a method widely employed in the system of psychology and sociology [27]. Narrative medicine, which combines narratology with medicine, was first proposed by Charan, which refers to a diagnosis and treatment activity carried out by doctors with narrative ability, whose core is empathy and reflection. At present, the definition of narrative nursing has not been unified. Some scholars have pointed out that narrative nursing is a nursing intervention method that applies narrative means to help patients reconstruct the meaning of disease stories [27]. Xiao defines the narrative practice as the composition of rewriting stories, recalling stories, reconstructing stories, reproducing brilliance, and externalizing stories, which are adopted to influence the narrator and the narrated [28]. Yang Yan defined narrative nursing as a nurse with the narrative ability to provide humane and effective nursing activities [29]. At present, narrative nursing refers to the nursing practice in that nurses help patients reconstruct the story of life and disease by listening, analyzing, and feedback from patients and find the starting point and main points of nursing and then intervening with the patients. In the process of narrative, guide patients to fully express their thoughts and vent their feelings through story narration, help patients specify the problems they face, make them look at them objectively, and give full play to their subjective initiative to actively construct new stories, so as to alleviate the pain [30]. At present, narrative nursing has been paid more attention by nursing professionals and carried out in clinical nursing practice, that is, through the use of various intervention measures, patients can carry out “disease narrative” in a variety of ways [31]. In some countries, patient narrative as a nursing method has been implemented in deathbed, elderly, and cancer patients and achieved good nursing results, such as in the study of Sunita and Deepika who carried out narrative nursing intervention in adult cancer patients [32]. The results indicated that the well-being index of cancer patients with the narrative nursing intervention was higher compared to the control group. They applied narrative nursing to mental nursing and found that the application of narrative nursing can help patients relieve mental tension and strengthen their psychological status [33].

Narrative nursing combined with thinking map health education has the following advantages: (1) through communication with patients, provide patients with the opportunity to talk to others to help patients release depression; meanwhile, analyze the causes of patients' depression and find the positive forces hidden behind negative emotions to reshape patients' self-cognition; (2) it can enhance the patients' self-confidence against the disease, thus improve the patients' sleep quality, reduce the patients' sense of insecurity and despair, enhance the patients' confidence, fully mobilize the patients' subjective initiative, enhance the patients' sense of self-worth, and improve patients' depression; (3) when patients talk about past positive events, they can not only give patients positive psychological hints but also make patients get a sense of well-being, which helps enhance their inner strength of patients; (4) in the process of implementing narrative nursing combined thinking map health education for patients, nurses and patients are in an equal cooperative relationship, and this relationship reduces patients' concerns to a certain extent, which is conducive to the communication between nurses and patients; (5) nursing staff in health education combined with some active treatment documents, as well as some letters and articles of special significance to patients, or can guide patients to better active treatment; these will also promote and guide patients to change their depression and enhance their self-confidence [34, 35].

RETRACTED

## 5. Conclusion

In this paper, we have focused our attention on finding a way to observe the effect of narrative nursing combined with thinking map health education on parturient self-efficacy and neonatal nursing ability. Experimental studies were carried out to verify the authenticity of our claim, and the results showed the idea is convincing. In the health education of primary parturient, the adoption of narrative nursing combined with thought guiding schema can enhance the level of nursing satisfaction and self-efficacy, strengthen the nursing ability of primiparas and the awareness rate of health knowledge, and reduce the occurrence of the maternal bad mood, which is more in line with the requirements of parturient.

## Figures and Tables

**Figure 1:** Comparison of the mastery of neonatal nursing ability.

**Figure 2:** Comparison of maternal health knowledge awareness score.

**Table 1:** Comparison of the score of maternal health knowledge awareness between the two groups [$\bar{x}\pm s$, points].

Group	*N*	Basic nursing of newborn	Physiological characteristics	Breastfeeding method	Environmental nursing knowledge	Vaccination and physical examination requirements

C group	30	12.59 ± 3.11	14.39 ± 2.34	15.38 ± 1.21	14.31 ± 2.44	12.49 ± 2.44
R group	30	20.63 ± 2.13	21.21 ± 1.22	19.59 ± 2.21	20.18 ± 2.15	19.59 ± 1.43
*t*		11.682	14.155	9.152	9.886	13.750
*P*		<0.01	<0.01	<0.01	<0.01	<0.01

RETRACTED

**Table 2:** Comparison of maternal self-efficacy between the two groups [$\bar{x}\pm s$, points].

Group	*N*	Promote development	Health care	Safety	Feeding	Total score

C group	30	56.38 ± 3.12	58.49 ± 4.44	62.39 ± 4.33	56.62 ± 5.23	63.51 ± 3.55
R group	30	73.31 ± 3.31	77.59 ± 3.73	77.19 ± 2.85	78.39 ± 3.31	76.59 ± 3.11
*t*		20.386	18.040	15.637	19.264	15.179
*P*		<0.01	<0.01	<0.01	<0.01	<0.01

**Table 3:** Comparison of anxiety and depression scores between the two groups [$\bar{x}\pm s$, points].

Group	*N*	Anxiety score		Depression score	
		Before nursing	After nursing	Before nursing	After nursing

C group	30	60.91 ± 3.12	52.91 ± 3.52	64.69 ± 1.67	54.23 ± 3.67
R group	30	60.93 ± 3.45	42.49 ± 3.11	64.94 ± 1.56	40.69 ± 3.56
*t*		0.023	12.150	0.599	14.504
*P*		>0.05	<0.01	>0.05	<0.01

## Data Availability

The data sets used and analyzed during the current study are available from the corresponding author upon reasonable request.
